# A Medical Image Registration Method Based on Progressive Images

**DOI:** 10.1155/2021/4504306

**Published:** 2021-07-27

**Authors:** Qian Zheng, Qiang Wang, Xiaojuan Ba, Shan Liu, Jiaofen Nan, Shizheng Zhang

**Affiliations:** Zhengzhou University of Light Industry, Zhengzhou, Henan 450002, China

## Abstract

**Background:**

Medical image registration is an essential task for medical image analysis in various applications. In this work, we develop a coarse-to-fine medical image registration method based on progressive images and SURF algorithm (PI-SURF) for higher registration accuracy.

**Methods:**

As a first step, the reference image and the floating image are fused to generate multiple progressive images. Thereafter, the floating image and progressive image are registered to get the coarse registration result based on the SURF algorithm. For further improvement, the coarse registration result and the reference image are registered to perform fine image registration. The appropriate progressive image has been investigated by experiments. The mutual information (MI), normal mutual information (NMI), normalized correlation coefficient (NCC), and mean square difference (MSD) similarity metrics are used to demonstrate the potential of the PI-SURF method.

**Results:**

For the unimodal and multimodal registration, the PI-SURF method achieves the best results compared with the mutual information method, Demons method, Demons+B-spline method, and SURF method. The MI, NMI, and NCC of PI-SURF are improved by 15.5%, 1.31%, and 7.3%, respectively, while MSD decreased by 13.2% for the multimodal registration compared with the optimal result of the state-of-the-art methods.

**Conclusions:**

The extensive experiments show that the proposed PI-SURF method achieves higher quality of registration.

## 1. Introduction

With the rapid development of computer technology and medical technology, medical images of different modalities can be obtained by means of computed tomography, nuclear magnetic resonance, and other imaging devices [1, 2]. In recent years, the image registration technique has been widely used in focus localization, patient rehabilitation, intraoperative guidance, and radiological diagnosis [3–8]. Medical image registration techniques draw more and more attention in clinical application.

Generally, the bulk of medical image registration techniques can be divided into two categories: intensity-based registration and feature-based registration [9–11]. Intensity-based registration plays an important role in the diagnosis and treatment of medical diseases. Since the end of the 20th century, researchers have proposed many related image registration algorithms. For example, Vercauteren et al. [12] developed the diffeomorphic Demons algorithm with a Lie group structure, which is computationally efficient. Maes et al. [13] proposed that mutual information could be used for medical image registration as a similarity measure. Ji [14] used the B-spline to refine the results after registering the medical image based on Demons. For feature-based medical image registration, firstly the feature points are extracted and matched; then, transformation parameters are obtained by calculating the matching relationship between the feature points, and finally, the registration between the images is completed. There are many classical feature matching algorithms. For example, Lowe developed a scale invariant feature transform (SIFT) method [15, 16]; Bay et al. proposed the speeded-up robust features (SURF) algorithm [17] by introducing an integral image to reduce the computation of feature points based on the SIFT method. The proposed algorithm not only has the advantages of SIFT in terms of image scaling and luminance variation but also reduces the computation of image feature points and shows excellent performance.

Compared with the popular deep learning-based registration methods in recent years, the above methods can be attributed to the traditional image registration technology. In the field of medical images, there are some common problems in deep learning-based methods [18], such as long training time, high requirement for hardware, and poor portability of model. The imprecision of the traditional registration method often appears due to the huge difference between floating image and reference image.

In this study, we developed a coarse-to-fine medical image registration method based on progressive images and SURF algorithm (PI-SURF) for higher registration accuracy. This method generates multiple progressive images combined with the SURF algorithm to extract features for further step-by-step registration. Unimodal and multimodal image registrations are given to verify the advantages of the PI-SURF method.

## 2. Evaluation Methods of Registration

A similarity measure is used to evaluate the result of image registration. During the registration process, the floating image is gradually aligned to the reference image, and the two images are most similar when the similarity measure is at the maximum/minimum. In this paper, we use the prevalent measures for quantitative evaluation of registration accuracy.

Mutual information (MI) is a measure of the degree of mutual dependence among random variables [19]. In this paper, it is used to evaluate the registration effect of reference image *R* and floating image *F*. The mutual information definitions of *R* and *F* are shown as

(1) $$\begin{array}{c} \text{MI}\left(R,F\right)=H\left(R\right)+H\left(F\right)-H\left(R,F\right),\\ H\left(R\right)=-\sum P_{R}\left(r\right)\log_{2}P_{R}\left(r\right),\\ H\left(F\right)=-\sum P_{F}\left(f\right)\log_{2}P_{F}\left(f\right),\\ H\left(R,F\right)=-\sum P_{RF}\left(r,f\right)\log_{2}P_{RF}\left(r,f\right), \end{array}$$

where *H*(*R*) and *H*(*F*) represent the information contained in the reference image *R* and the floating image *F*, respectively; *P*_*R*_(*r*) and *P*_*F*_(*f*) are the marginal probability distribution; *P*_*RF*_(*r*, *f*) is the joint probability distribution; and *H*(*R*, *F*) is the joint entropy of *R* and *F*.

Normalized mutual information (NMI) is an expression to measure the degree of similarity of two images [20]. The larger the value of NMI, the higher the similarity of two images. It is usually used as an evaluation index in image registration and is given by

(2) $$\begin{array}{c} \text{NMI}\left(R,F\right)=\frac{H\left(R\right)+H\left(F\right)}{H\left(R,F\right)}. \end{array}$$

The normalized correlation coefficient (NCC) is useful for image registration [21] and is in the range of [0, 1]. The formula is shown as

(3) $$\begin{array}{c} \text{NCC}\left(R,F\right)=\frac{\sum_{x=1}^{m}\sum_{y=1}^{n}\left(R\left(x,y\right)-\bar{R}\right)\left(F\left(x,y\right)-\bar{F}\right)}{\sqrt{\sum_{x=1}^{m}\sum_{y=1}^{n}{\left(R\left(x,y\right)-\bar{R}\right)}^{2}}\sqrt{\sum_{x=1}^{m}\sum_{y=1}^{n}{\left(F\left(x,y\right)-\bar{F}\right)}^{2}}}, \end{array}$$

where *R*(*x*, *y*) and *F*(*x*, *y*) are the intensity of the pixel (*x*, *y*) in the reference image *R* and the floating image *F*, respectively; $\bar{R}$ and $\bar{F}$ are the mean of the reference image *R* pixels and the floating image *F* pixels, respectively; and *m*∗*n* is the size of the image.

Mean square difference (MSD) is a similarity measure based on the gray difference between a reference image and a floating image [22]. When the two images are the most similar, the mean square deviation is the smallest. Mathematically, the definition is described by

(4) $$\begin{array}{c} \text{MSD}=\frac{\sum_{x=1}^{m}\sum_{y=1}^{n}{\left(R\left(x,y\right)-F\left(x,y\right)\right)}^{2}}{N}, \end{array}$$

where *N* is the total number of pixels in the image.

## 3. Methods

Extracting the feature points from floating image *F* and reference image *R* is needed firstly in image registration, and the coordinates of matching point pairs of the images to be registered are obtained with establishing the mapping relation between the two images and estimating the parameters of affine transformation. Then, the floating image is transformed to the same coordinate space with the reference image. Finally, the bicubic interpolation algorithm is used to reassign the floating image to perform the whole registration process. Despite the excellent performance of the SURF algorithm, there is still a problem of low registration accuracy. The reason for this phenomenon is that the algorithm operates directly on the original image, usually contaminated by the environment which leads to poor quality of the images, so it is difficult to extract the feature, which leads to the decrease of the number and accuracy of the effective feature points. In order to solve the problem of large structure difference between medical images to be registered, we attempt to generate intermediate progressive images for a coarse-to-fine registration. The proposed PI-SURF, including six main elements: generating the intermediate progressive images, SURF feature points detection and description, point matching, bicubic interpolation, the coarse registration, and the fine registration, can be implemented in the following steps.

**Step 1 .**

Average each corresponding pixel of the floating image *F* to be registered and the reference image *R*, and the resulting image is a progressive image *M*_0_ between the two images. The calculation formula is shown as

(5) $$\begin{array}{c} M_{0}\left(x,y\right)=\frac{F\left(x,y\right)+R\left(x,y\right)}{2}. \end{array}$$

**Step 2 .**

Repeat Step 1 with intermediate progressive image *M*_0_, floating image *F* to be registered, and reference image *R* to generate intermediate progressive images *M*_1_, *M*_2_, ⋯, *M*_*l*_. The intermediate progressive image *M*_*l*_ is selected iteratively as the reference image in the intermediate registration process.

**Step 3 .**

Feature points are extracted from floating image *F* to be registered and intermediate progressive image *M*_*l*_. It is well known that the value of the pixel in the rectangle can be quickly calculated by using the integral image in the SURF algorithm. With the help of the integral image, the Gauss filtering of the image is transformed into addition and subtraction operation of the integral image, which can significantly improve the calculation speed.

The corresponding value of the integral image is defined as

(6) $$\begin{array}{c} I_{\sum }\left(x,y\right)=\underset{x^{\prime }\leq x,y^{\prime }\leq y}{\sum }I\left(x^{\prime },y^{\prime }\right). \end{array}$$

At the same time, the Hessian matrix is used to extract feature points, and each pixel of the image has a corresponding Hessian matrix, which is defined as

(7) $$\begin{array}{c} H\left(x,y,\sigma \right)=\left[\begin{array}{cc} L_{xx}\left(x,y,\sigma \right) & L_{xy}\left(x,y,\sigma \right)\\ L_{xy}\left(x,y,\sigma \right) & L_{yy}\left(x,y,\sigma \right) \end{array}\right], \end{array}$$

where *L*_*xx*_(*x*, *y*, *σ*) is the convolution of the Gaussian second-order derivative *∂*^2^/*∂x*^2^*g*(*x*, *y*, *σ*) with the image *F* in the *x* direction and similarly for *L*_*xy*_(*x*, *y*, *σ*) and *L*_*yy*_(*x*, *y*, *σ*). A two-dimensional Gaussian kernel function is defined as

(8) $$\begin{array}{c} g\left(x,y,\sigma \right)=\frac{1}{2{\pi \sigma }^{2}}\exp\left(-\frac{x^{2}+y^{2}}{2\sigma^{2}}\right), \end{array}$$

where *σ* is the scale factor. It is important for constructing the Hessian matrix to generate stable edge points of the image. The image needs to be smoothed by Gauss filter to eliminate interfering noise prior to constructing the Hessian matrix, and then, the second derivative is obtained, which is a contribution to locate the key points that are brighter or darker than the other points in the surrounding area. In the SURF algorithm, in order to keep the size of the image unchanged, an image pyramid is constructed by using the scaling-up box filter and convolution to form the scale space. Each pixel processed by the Hessian matrix is compared with the 26 pixels in the neighborhood of the scale space for locating the key points preliminarily. The nonmaximum suppression is followed to eliminate key points with weak energy and false located in order to preserve the final stable feature points.

**Step 4 .**

Establish the database of image feature points, where the data structure includes position coordinates, scale, direction, and feature vector, which is useful for matching each feature point of the image in the database one by one. The Euclidean distance of the feature vector, namely, matching degree, is calculated to find the first nearest neighbor and the next nearest neighbor feature points in the database. The feature points of the floating image *F* and the intermediate progressive image *M*_*l*_ are *x* = (*x*_1_, *x*_2_, ⋯, *x*_*t*_) and *x*′ = (*x*_1_′, *x*_2_′, ⋯, *x*_*t*_′), respectively. The Euclidean distance is computed according to

(9) $$\begin{array}{c} \text{dist}=\sqrt{\overset{n}{\underset{t=1}{\sum }}{\left(x_{t}-{x_{t}}^{\prime }\right)}^{2}}. \end{array}$$

**Step 5 .**

The space transformation of the floating image *F* is performed by using the affine transformation of the bicubic interpolation. The affine transformation is essentially a simple superposition of the linear transformation and the translation transformation, and its basic transformations mainly include scaling, translation, rotation, reflection, and skew. Affine transformation is an important transformation method in a two-dimensional plane, which is widely used in image registration. In two-dimensional image transformation, the general expression is given by

(10) $$\begin{array}{c} \left[\begin{array}{c} x\\ y\\ 1 \end{array}\right]=\left[\begin{array}{ccc} R_{00} & R_{01} & T_{x}\\ R_{10} & R_{11} & T_{y}\\ 0 & 0 & 1 \end{array}\right]\left[\begin{array}{c} x^{\prime }\\ y^{\prime }\\ 1 \end{array}\right]. \end{array}$$

The obtained parameters are transformation parameters *R*_00_, *R*_01_, *R*_10_, *R*_11_ and displacement parameters *T*_*x*_, *T*_*y*_. *x*, *y*, and *x*′, *y*′ are the coordinates of the corresponding matching points in the reference image *R* and the floating image *F*. The initial coarse image registration result is obtained by applying the obtained parameters to the floating image.

**Step 6 .**

Repeat Steps 3–5 with the reference image and the initial coarse image registration result to further get the fine registration result.

**Step 7 .**

Repeat Steps 3–6 to get the best registration results with the optimal progressive image.

The mentioned above process of the proposed PI-SURF method can be illustrated in Figure 1.

## 4. Experiments and Results

In this study, the progressive image selection, the matching experiments of feature points from two images, unimodal MR-MR, and multimodal CT/MR medical image registration were carried out to verify the accuracy and validity of the proposed algorithm. The unimodal MR-MR images are from the Brainweb database of the Monte Neuromedicine Department (https://brainweb.bic.mni.mcgill.ca/). This article randomly selects 20 groups of brain two-dimensional slice images (T1- and PD-weighted MR images), the size is 181∗217, the slice thickness is 1 mm, and the noise level is 0%. The multimodal CT/MR images are given by the official Kaggle (https://www.kaggle.com/vbookshelf/computed-tomography-ct-images and https://www.kaggle.com/navoneel/brain-mri-images-for-brain-tumor-detection), of which 20 groups are selected randomly and the image size is 225∗225.

The registration results were evaluated by four similarity measures, including MI, NCC, MSD, and NMI. The higher the values of mutual information, normalized correlation coefficient, and normalized mutual information, the better the registration effect of the reference image and floating image. The experiments were implemented on a desktop computer with an Intel® Core™ I79750h CPU, 32 GB of RAM using MATLAB R2019a version. The developed algorithm is compared with the state-of-the-art registration algorithms, including the mutual information algorithm [13], Demons algorithm [12], Demons+B-spline algorithm [14], and SURF algorithm [17], to show the promising results.

### 4.1. Progressive Image Selection

The first experiment was designed to demonstrate the appropriate progressive image for the best registration results.  Figure 2 illustrates the performance of the progressive image on the registration results, and *M*_7_ is the optimal progressive image. As more intermediate images are generated, the effect of edge feature points obtained by initial registration is less ideal, which affects the choice of space transformation parameters, leading to the inaccurate result of image registration. In this study, we choose *M*_7_ as the progressive image in the following experiments.

### 4.2. Image Feature Point Matching

Feature points are extracted from the floating image and reference image using the SURF algorithm. The direct matching of the feature points between the reference image and the floating image is shown in Figure 3(a). The matching effect of feature points based on the proposed progressive images is shown in Figures 3(b) and 3(c).  Table 1 presents the feature point matching results. The SURF method obtains 30 matching pairs of feature points between the floating image and the reference image, of which 16 pairs are mismatched and 14 pairs are correctly matched with 47% accuracy. There are 30 matching pairs between floating image and intermediate progressive image in the coarse registration stage, including 7 pairs of mismatching feature points and 23 pairs of correct matching feature points, reaching 77% accuracy. There are 29 pairs of matching feature points for fine registration, achieving 55% accuracy. The PI-SURF reduces the error rate of the feature points and will improve the accuracy of the whole image registration as expected.

### 4.3. Unimodal Registration Results

The T1-weighted MR image is selected as the floating image *F*, and the PD-weighted MR image is selected as the reference image *R* as shown in Figure 4. The golden standard contrast maps used in the experiment are all the images that have been registered by the medical experts manually. Each algorithm is tested 100 times, and the average values of mutual information, normalized correlation coefficient, mean square deviation, and normalized mutual information are calculated. Figures 4(c)–4(g) are the registration results of floating images based on the mutual information algorithm, Demons algorithm, Demons+B-spline algorithm, SURF algorithm, and PI-SURF algorithm.

Table 2 presents the unimodal registration results based on various registration methods. In general, compared with the Demons algorithm and Demons+B-spline algorithm, the mutual information, normalized correlation coefficient, and normalized mutual information of the PI-SURF algorithm are improved, and the mean square difference is reduced to 0.0082.

### 4.4. Multimodal Registration Results

Figure 5(a) is a MR image as the floating image, and Figure 5(b) is a CT image as the reference image, respectively. Figures 5(c)–5(g) are the registration results of the floating image based on the mutual information algorithm, Demons algorithm, Demons+B-spline algorithm, SURF algorithm, and PI-SURF algorithm.

Table 3 shows the average values of 100 registration experiments using MI, NCC, MSD, and NMI as the measure functions for reference images and floating images. The results show that the proposed algorithm is better than the other four algorithms in terms of MI, NCC, MSD, and NMI.

## 5. Discussion

It is obvious that the developed PI-SURF method is more accurate than other registration methods. In this section, we firstly discuss the impact of the registration mechanism based on the progressive image and then discuss the difference between the proposed algorithm and the existing state-of-the-art registration algorithms. The key of the developed algorithm is that the progressive registration mechanism is utilized to reduce the difference between the floating image and the reference image. As shown in Figure 3(a), the floating image is registered directly to the reference image, and the matching pairs of corresponding feature points obtained from the two images are less and the matching accuracy is lower. This phenomenon is because the SURF algorithm performs the feature matching of two images by calculating the extreme point in the image and using it as the feature point. Some feature points cannot be detected in the process. For example, dark spots in bright areas or bright spots in dark areas cannot be detected by the SURF algorithm, resulting in the loss of some key image feature points. In addition, many feature points in the floating image are matched to the same feature point of the reference image, indicating that the transformation parameters are not accurate and the accuracy of registering two images is greatly reduced. The proposed PI-SURF method uses the intermediate progressive image to register the floating image firstly and finds more edge feature points, which can improve the image edge matching as shown in Figure 3(b). The initial coarse registration image and the reference image are used for fine registration to reduce the error rate of the feature points and improve the accuracy of the whole image registration. Compared with the direct registration from the floating image to the reference image, the mismatching pairs of feature points in the coarse registration decrease by 9, and the rate of correct matching pair increases by 30%. For the fine registration, the number of matching pairs of feature points decreases, but the number of correct matching pairs increases, and the rate of correct matching increased by 8%. Moreover, compared with the direct registration between two images, the proposed coarse-to-fine registration using the progressive image can avoid the situation to a certain extent where multiple feature points are matched to the same feature point, while providing reliable coordinates for subsequent spatial transformations.

The mutual information algorithm is to calculate the entropy of two images, measuring the degree of mutual inclusion of information between them. The bigger the mutual information between two images, the better the result of image registration. However, mutual information is sensitive to the overlap area between two images. When the overlap area of two images is too small, mutual information is small, and the registration accuracy decreases. The Demons algorithm and Demons+B-spline algorithm are based on the principle of gray-scale conservation of two images, while multimodal images cannot simply use gray-scale conservation to calculate driving force. The SURF algorithm is a registration algorithm based on image features, which has the characteristics of high efficiency and can save registration time effectively. However, the SURF algorithm is unstable when searching for feature points and matching between point pairs, and it is easy to make more mismatches, which will influence the accuracy of registration. In this paper, progressive registration can guarantee the accuracy of image registration.

It is noticed that there are several limitations in the study of this paper. Firstly, many intermediate progressive images are generated at the cost of time to some extent. Secondly, in the PI-SURF registration mechanism, there is still mismatching after extracting and matching the image feature points due to the SURF algorithm. Thirdly, the proposed algorithm is only tested on two-dimensional human brain images. Future studies are warranted to introduce the algorithm of eliminating mismatching points to further increase the correct rate of matching points and extend the PI-SURF to register the three-dimensional human brain images.

## 6. Conclusions

To solve the problem of low registration accuracy of traditional medical image registration algorithms, this paper presents a medical image registration algorithm based on progressive images and SURF algorithm from coarse to fine. Multiple intermediate progressive images are generated, and the SURF algorithm is used to perform the two-stage image registration. The idea, progressive images, and coarse-to-fine registration can be extended to other registration algorithms. The extensive experiments show that the image registration based on intermediate progressive presented in this paper has a good improvement compared with the state-of-the-art algorithms, which can be used for medical image registration in clinical application.

## Figures and Tables

**Figure 1:** The flowchart of the proposed method.

**Figure 2:** The registration results with the various progressive images.

**Figure 3:** Image feature point matching based on progressive image.

**Figure 4:** Comparison of unimodal registration results.

**Figure 5:** Comparison of multimodal registration results.

**Table 1:** Comparison of feature point matching.

Algorithm	Feature points	Correct feature points
SURF	30	14
PI-SURF (coarse registration)	30	23
PI-SURF (fine registration)	29	16

**Table 2:** Comparison of experimental results of unimodal image registration.

Method	Evaluation index			
	MI	NCC	MSD	NMI
Mutual information	1.4394	0.7703	0.0710	1.1149
Demons	2.0726	0.8389	0.1054	1.1971
Demons+B-spline	2.0845	0.6617	0.1094	1.1978
SURF	1.7156	0.8142	0.0197	1.1559
PI-SURF	2.2577	0.9219	0.0082	1.2161

**Table 3:** Comparison of experimental results of multimodal image registration.

Method	Evaluation index			
	MI	NCC	MSD	NMI
Mutual information	1.3172	0.6543	0.0695	1.1617
Demons	1.2712	0.6634	0.0677	1.1559
Demons+B-spline	1.3255	0.6837	0.0632	1.1609
SURF	1.3733	0.5847	0.06	1.1539
PI-SURF	1.5861	0.7334	0.0521	1.1769
